The article "Determination of the Efficiency of Magnetic Resonance Imaging in the Evaluation of Compressive Myelopathy" was retracted in 2024. Reasons: plagiarized images; overlap with other authors' work.

# Determination of the Efficiency of Magnetic Resonance Imaging in the Evaluation of Compressive Myelopathy

**DOI:** 10.7759/cureus.57874

**Published:** 2024-04-08

**Authors:** Challa Anil Kumar, Satyanarayana Kummari, Bagadi Lava Kumar

**Affiliations:** 1 Department of Radiodiagnosis, Great Eastern Medical School & Hospital, Srikakulam, Andhra Pradesh, IND; 2 Department of Radiodiagnosis, All India Institute of Medical Sciences, Nagpur, Maharashtra, IND

**Keywords:** mri, compressive myelopathy, spinal cord, traumatic myelopathy, spondylitis, pott’s spine, metastases, extradural lesions, intradural lesions, epidural abscess

## Abstract

Background

The phrase "compressive myelopathy" refers to compression of the spinal cord, either internally or externally. This compression might arise from various sources such as a herniated disc, post-traumatic compression, and epidural abscess as well as epidural or intradural neoplasms. Magnetic resonance imaging (MRI) plays a crucial role in differentiating between compressive and non-compressive myelopathy. After eliminating compressive lesions, attention is directed toward intrinsic cord-related causes of acute myelopathy including vascular, infectious, and inflammatory pathologies.

Aims

The study aimed to assess different etiologies of compressive myelopathy, analyze the MRI features of spinal cord compressive lesions, classify the lesions depending on site, and correlate MRI findings with intraoperative findings and histopathology in operated cases.

Material & methods

A total of 50 patients, who exhibited clinical symptoms indicative of compressive myelopathy sent to the Radiology department, Rangaraya Medical College (RMC), Kakinada for MRI spine were included in the study. It’s an observational cross-sectional study. Statistical Package for Social Sciences (SPSS) version 22.0 (IBM Corp., Armonk, USA) was used for statistical calculations.

Result

Among the 50 cases of compressive myelopathy, the etiologies are distributed as follows: trauma (22 cases), infection (12 cases), primary neoplasm (eight cases), and secondary neoplasm (eight cases); extradural compressive lesions (84%) and Intradural-extramedullary lesions (16%).

Conclusion

Utilizing MRI successfully assessed the spinal cord integrity and characterized spinal tumors. Consequently, the study concludes that MRI is a highly definitive, sensitive, and accurate tool for evaluating compressive myelopathy.

## Introduction

Compressive myelopathy refers to the compression of the spinal cord, which can occur either externally or internally within the cord itself. This compression might arise from various sources such as a herniated disc, post-traumatic compression resulting from fractures or displaced vertebrae, epidural hemorrhage or abscess, as well as epidural or intradural neoplasms which can be extramedullary or intramedullary. The common benign extradural masses are degenerative and traumatic lesions such as disc herniation, osteophytes, and fractures, and the common malignant extramedullary intradural tumours are spinal leptomeningeal metastases and non-Hodgkin lymphoma [1].

The article "Determination of the Efficiency of Magnetic Resonance Imaging in the Evaluation of Compressive Myelopathy" was retracted in 2024. Reasons: plagiarized images; overlap with other authors' work.

Magnetic resonance imaging (MRI) is the only currently available technique that provides direct visualization of the spinal cord. The ability of MRI to show the spine and spinal cord with greater sensitivity and specificity than myelography and CT scan is well established for trauma, neoplastic, congenital, and degenerative diseases. Plain radiographs are limited in their ability to detect traumatic spinal lesions with high sensitivity. MRI is the primary imaging method for evaluating soft tissue injuries in the spine, particularly for assessment of the spinal cord, intervertebral discs, and posterior elements. It also enables the differentiation of spinal epidural hematoma, spinal cord haemorrhage, and edema, which can hold prognostic significance. MRI imaging reveals the connection between fractured or misaligned vertebrae and the spinal cord while highlighting significant narrowing of the spinal canal. Signal irregularities within the spinal cord can be detected, aiding in the precise localization and determination of the extent of the trauma [2, 3].

Accurate and timely diagnosis of infective spondylodiscitis is crucial, as missed or delayed diagnosis can potentially lead to the development of paraspinal, psoas muscle abscesses, epidural abscesses, and spinal cord compression, along with vertebral body destruction and spinal instability. MRI is the imaging modality of choice due to its very high sensitivity and specificity. It is also useful in differentiating between pyogenic, tuberculous, and fungal infections, and a neoplastic lesion [1].

When there is suspicion of cord compression caused by a neoplasm, MRI stands out as an excellent imaging technique for visualizing tumors that affect the spine. Currently, MRI is regarded as the preferred method for the comprehensive assessment of spinal neoplasms. These neoplasms are typically classified based on their location as extradural, intradural, or intramedullary [4, 5]. Within the extradural space, a variety of primary bone tumors can arise, although the occurrence of most primary bone tumors is uncommon, with some exceptions like hemangioma. Metastases, on the other hand, are more frequently observed in the extradural space [6]. Primary tumours such as neurofibroma and meningioma are frequently found in the intradural extramedullary space. In the past, leptomeningeal metastases or secondary tumours were thought to be extremely uncommon. Nevertheless, it is being observed more frequently. The current rise in leptomeningeal tumors can be attributed to both enhanced diagnostic capabilities and a genuine rise in their occurrence. Primary tumours are far more common than metastases inside the intramedullary region [7].

The article "Determination of the Efficiency of Magnetic Resonance Imaging in the Evaluation of Compressive Myelopathy" was retracted in 2024. Reasons: plagiarized images; overlap with other authors' work.

MRI is essential for distinguishing between compressive and non-compressive myelopathy. After eliminating compressive lesions, attention is directed towards intrinsic cord-related causes of acute myelopathy, including vascular, infectious, and inflammatory pathologies. Swift recognition and treatment of many spinal cord diseases at an early stage are crucial for potential reversibility, making them some of the most critical neurological emergencies [8, 9].

To our knowledge, there are only a few comprehensive studies in the literature evaluating various etiologies of compressive myelopathy, analyzing the MRI features of the lesions, classifying the lesions, and correlating the MRI findings with surgical, cytological, and histopathological results.

The research aimed to evaluate various etiologies of compressive myelopathy, analyze the MRI features of spinal cord compressive lesions, classify the lesions as extradural or intradural based on their location, and establish a correlation between MRI findings, intraoperative observations, cytological and histopathological results in operated cases. This correlation will contribute towards validating the diagnostic accuracy and predictive value of MRI in assessing spinal cord compressive lesions, thereby enhancing our understanding of their clinical implications and informing appropriate treatment strategies.

## Materials and methods

It was an observational cross-sectional prospective study. A total of 50 patients, who exhibited clinical symptoms indicative of compressive myelopathy referred to the radiology department at Rangaraya Medical College (RMC), Kakinada, India for MRI spine were included in the research. The duration of the study was 2 years. Every patient involved in the research gave their informed assent. The research received permission from the institutional ethics committee.

Inclusion criteria

All the patients, who exhibited clinical symptoms indicative of compressive myelopathy referred to the radiology department for MRI spine, were included in the research.

Exclusion criteria

Patients with non-compressive myelopathy, disc herniation, patients who were contraindicated to undergo MRI, and patients who did not assent to be a part of the research were excluded from the research. 

The article "Determination of the Efficiency of Magnetic Resonance Imaging in the Evaluation of Compressive Myelopathy" was retracted in 2024. Reasons: plagiarized images; overlap with other authors' work.

MR image acquisition

General Electric (GE, Boston, USA) 1.5 Tesla MRI Electromagnet Version: Conventional surface and body coils were utilized for the acquisition of images of the cervical, thoracic, and lumbar spine. MRI sequences used and their parameters are listed in Table 1.

**Table 1:** MRI sequences and their parameters SE T1 WI: Spin echo T1 weighted imaging; FSE T1 WI: Fast spin echo T1 weighted imaging; T2 WI: T2 weighted imaging; GRE: Gradient echo; STIR: Short tau inversion recovery

Sequences	Repetition time (msec)	Echo time (msec)	Flip angle
SE T1 WI	500	23	70°
FSE T1 WI	440	14	90°
T2 WI	3000	120	90°
GRE	612-1000	27	30°
STIR	4400	20	90°

Technique

The patients underwent MRI scans while lying down, with the body adequately placed and immobilized. Conventional surface coils were utilized for image acquisition. Sagittal T1 weighted imaging (T1WI), T2 weighted imaging (T2WI), Short tau inversion recovery (STIR), Axial T1WI, T2WI, Axial Gradient echo (GRE), post-contrast T1WI axial, sagittal, and coronal sequences were routinely obtained. Contrast was not used in cases with spinal trauma. Neuroradiologists with a minimum of five years of experience in the field assessed the various etiologies of compressive myelopathy, analyzed the MRI features of spinal cord compressive lesions, and classified the lesions as extradural or intradural based on their location. MRI findings were correlated with intraoperative observations and cytological and histopathological results in operated cases.

Statistical analysis

Statistical computations were performed using Statistical Package for Social Sciences (SPSS) for Windows, version 22.0 (IBM Corp., Armonk, USA).

## Results

In the current research, a significant proportion of patients with spinal trauma (n=8)(36.36%) and primary neoplasms (n=5)(62.5%) belong to middle age (20-49 years). The majority of patients diagnosed with spinal infection (n=5)(41.66%) and metastases (n=6)(75%) were in the older age group (>50 years). The majority of spinal traumas (n=19)(86.36%) occurred in males, but spinal infections (n=7)(58.33%), primary neoplasms (n=5)(62.5%), and secondary neoplasms (n=5)(62.5%) were more prevalent in females. Extradural compression was most frequently caused by spinal trauma and infection, whereas primary neoplasms were more frequently found in the intradural compartment. Age, gender, and location dispersion of different lesions are listed in Table 2.

**Table 2:** Age, gender, and location dispersion of different lesions

MRI Diagnosis				
Age (in Years)	Traumatic n(%)	Infection n(%)	Primary Neoplasm n(%)	Metastases n(%)
12-30	7(31.8%)	3(25%)	0(0%)	0 (0%)
31-50	8(36.36%)	4(33.3%)	5(62.5%)	2(25%)
>50	7(31.8%)	5(41.66%)	3(37.5%)	6(75%)
Gender				
Male	19(86.36%)	5(41.66%)	3(37.5%)	3(37.5%)
Female	3(13.63%)	7(58.33%)	5(62.5%)	5(62.5%)
Location				
Extradural	22(100%)	12(100%)	0 (0%)	8(100%)
Intradural	0(0%)	0(0%)	8(100%)	0(0%)

Out of the 50 cases, trauma was observed in 22 cases, infection in 12 cases, primary neoplasms in eight cases, and secondary neoplasms in eight cases (Table 2, 3). The primary etiology of compressive myelopathy in the current research was spinal trauma (n=22)(44%) followed by spinal infection (n=12)(24%). The most frequent etiology of compressive myelopathy was extradural compressive lesions (n=42)(84%), which are followed by intradural-extramedullary lesions (n=8)(16%). Etiologies of compressive myelopathy are listed in Table 3.

The article "Determination of the Efficiency of Magnetic Resonance Imaging in the Evaluation of Compressive Myelopathy" was retracted in 2024. Reasons: plagiarized images; overlap with other authors' work.

**Table 3:** Etiologies of compressive myelopathy

Etiologies	No. of cases (n=50)	Percentage (%)
Traumatic Myelopathy	22	44
Infection	12	24
Primary neoplasm	8	16
Metastases	8	16

Out of the 22 patients with spinal trauma, the most common cause of injury was a road traffic accident which accounted for 70% of the cases, while falls from height accounted for the remaining 30%. The distribution of injuries occurred at the thoracic level (54.4%), followed by cervical (36.36%), and lumbar (9.1%) levels. Spinal cord compression was demonstrated in all 22 patients with spinal trauma. Vertebral body subluxation was seen in 12 cases and epidural hematoma in 10 cases. The MRI revealed signal alterations in the spinal cord in all patients. Additionally, posterior element fractures were found in seven patients, ligamentous disruption in seven patients, soft tissue injuries in six patients, and epidural hematomas in six patients (Figure 1).

**Figure 1:** Traumatic myelopathy Sagittal T2 weighted images (A, B) of the cervical spine show grade IV anterolisthesis of C6 over C7 vertebra with T2 hyperintensities in the spinal cord at C2-D1 level and severe spinal cord compression. Intraoperative image (C) and post-operative radiograph (D).

In the current research, culture and sensitivity, cytology and histopathology revealed 12 cases of spinal infection (Table 3). Among them, eight cases in the thoracic spine and four cases in the lumbar spine. MRI revealed the destruction of the vertebral bodies along with the presence of pre and paravertebral collections in eight cases. All 12 cases showed a compressed spinal cord due to an epidural component (Figures 2, 3).

**Figure 2:** Epidural abscess Contrast-enhanced cervicodorsal Sagittal T1 weighted (A) and dorsolumbar Sagittal T1 weighted (B), cervicodorsal Sagittal T2 weighted (C), and post-contrast Axial T1 weighted (D) images of the spine show an elongated peripherally enhancing collection with extensive posterior epidural extension.

The article "Determination of the Efficiency of Magnetic Resonance Imaging in the Evaluation of Compressive Myelopathy" was retracted in 2024. Reasons: plagiarized images; overlap with other authors' work.

**Figure 3:** Koch’s spine with prevertebral and paravertebral collections Sagittal T1W (A) and T2W (B), Axial T2W (C) and Coronal STIR (D) images of the dorsal spine show T1 and T2 heterogeneous signal intensities in the involved dorsal vertebrae with prevertebral and paravertebral collections as well as consolidations and cavitary lesions in bilateral upper lobes (Right>>Left). T1W: T1 weighted; T2W: T2 weighted; STIR: Short tau inversion recovery

Four cases were found to be related to cord edema. Mycobacterium tuberculosis was the most common organism responsible for spinal infection causing compressive myelopathy. Types of infection are listed in Table 4.

**Table 4:** Types of infection

Type of infection	No. of Patients (n=12)	Percentage (%)
Tuberculosis	8	66.6
Pyogenic infections	4	33.3
Fungal infections	0	0.0
Total	12	100

In the current research, there were eight (16.7%) cases of primary intradural extramedullary tumours. Among these cases, five were identified as neurofibromas and three as meningiomas on histopathology (Tables 5, 6). Among the neurofibromas, MRI diagnosed three cases as neurofibromas and two cases equivocal between neurofibroma and meningioma (Figures 4, 5). 

**Table 5:** Incidence and location of the primary neoplasms

Primary neoplasms	No. of patients (n=8)	Cervical	Thoracic	Lumbar
Neurofibroma	5	3	2	0
Meningioma	3	0	2	1
Total	8	3	4	1

**Table 6:** Correlation of MRI diagnosis with cytology and histopathology

Diagnosis	MRI (n=50)	Cytology and Histopathology	% correlation
Traumatic Myelopathy	22	-	-
Infection	12	10	83.3
Metastases	8	8	100.0
Neurofibroma	5	3	60.0
Meningioma	3	2	66.6

**Figure 4:** Neurofibroma Sagittal T1W (A) and T2W (B), contrast-enhanced Axial T1W (C), and Sagittal T1W (D) images of the cervical spine show T1 isointense and T2 hyperintense intradural lesion at C3-C4 level with homogeneous enhancement on post contrast study. T1W: T1 weighted; T2W: T2 weighted.

**Figure 5:** Neurofibroma Sagittal T1W (A) and T2W (B), post-contrast Coronal T1W (C) and Sagittal T1W (D) images of the cervical spine show T1 hypointense and T2 hyperintense intradural lesion at C1-C2 level with enhancement on contrast study. T1W: T1 weighted; T2W: T2 weighted.

Among the meningiomas, MRI diagnosed one case as meningioma and two cases as equivocal between meningioma and neurofibroma. Meningiomas frequently occurred in the thoracic region, but neurofibromas were frequently found in both the thoracic and cervical regions (Figures 6, 7). The incidence and location of the primary neoplasms are listed in Table 5.

The article "Determination of the Efficiency of Magnetic Resonance Imaging in the Evaluation of Compressive Myelopathy" was retracted in 2024. Reasons: plagiarized images; overlap with other authors' work.

**Figure 6:** Meningioma Sagittal T1W (A) and T2W (B), contrast-enhanced Axial T1W (C) and Sagittal T1W (D) images of the dorsal spine show T1 isointense and T2 iso to hypointense intradural lesion with post-contrast enhancement. T1W: T1 weighted; T2W: T2 weighted.

**Figure 7:** Meningioma Sagittal T1W (A) and T2W (B), contrast-enhanced Axial T1W (C) and Sagittal T1W (D) images of the dorsal spine show T1 and T2 isointense intradural lesion with homogeneous enhancement and dural tail sign on post contrast study. T1W: T1 weighted; T2W: T2 weighted.

In the current research, there were eight (16.7%) cases of spinal metastases on histopathology (Table 6). Cord compression in all eight patients was caused by intraspinal extradural masses originating from an aberrant portion of the vertebra. Five (62.5%) of the eight participants had multiple lesions. The most prevalent location for spinal metastases was the thoracic region (n=4)(50%) followed by the cervical (n=2)(25%) and lumbar region (n=2)(25%). There were three cases of carcinoma of the bronchus (Figure 8), three cases of carcinoma of the breast, one case of lymphoma, and one case of carcinoma of the prostate (Figure 9). The correlation of MRI diagnosis with cytology and histopathology is given in Table 6.

**Figure 8:** Metastasis from carcinoma bronchus Sagittal T1W (A), T2W (B), and Axial T1W (C) images of the cervical spine show T1 and T2 hypointense lesion in the C7 vertebra with epidural component. T1W: T1 weighted; T2W: T2 weighted.

**Figure 9:** Sclerotic metastasis from carcinoma prostate Sagittal T1W (A), T2W (B) and Axial T1W (C) images of the cervicodorsal spine show T1 and T2 hypointense lesion in the D8 vertebra with epidural component. T1W: T1 weighted; T2W: T2 weighted.

## Discussion

The widely acknowledged superiority of MRI lies in its heightened sensitivity and specificity as compared to myelography and computed tomography scan (CT) for visualizing the spine in cases of trauma, and neoplastic, congenital, and degenerative diseases. Notably, MRI stands as the sole available technique enabling precise imaging of the spinal cord. Furthermore, its capability for precise soft tissue definition and non-invasive nature has solidified its prominence. MRI sequences used and their parameters are listed in Table 1.

Out of the 50 cases, trauma was observed in 22 cases, infection in 12 cases, primary neoplasms in eight cases, and secondary neoplasms in eight cases (Table 2, 3). Out of the 22 patients with spinal trauma, the most common cause of injury was a road traffic accident which accounted for 70% of the cases, while falls from height accounted for the remaining 30%. According to research performed by Kulkarni et al. the most frequent cause of spinal cord injury was road traffic accidents, while falls were the least prevalent cause [10, 11]. The type of trauma in the present study yielded comparable findings.

The article "Determination of the Efficiency of Magnetic Resonance Imaging in the Evaluation of Compressive Myelopathy" was retracted in 2024. Reasons: plagiarized images; overlap with other authors' work.

The distribution of injuries occurred at the thoracic level (54.4%), followed by cervical (36.36%), and lumbar (9.1%) levels. This distribution aligns with the findings from research performed by Kerslake et al. [12].

Spinal cord compression was demonstrated in all 22 patients with spinal trauma. Vertebral body subluxation was seen in 12 cases and epidural hematoma in 10 cases. The MRI revealed signal alterations in the spinal cord in all patients. Additionally, posterior element fractures were found in seven patients, ligamentous disruption in seven patients, soft tissue injuries in six patients, and epidural hematomas in six patients (Figure 1). In the current study, the intraoperative findings were juxtaposed with the results from MRI and concluded that MR imaging exhibits sensitivity in detecting injuries to the disc, posterior longitudinal ligament, and interspinous ligament/soft tissues. This aligns with the conclusions reported in the research conducted by Kulkarni et al. and Goradia D et al. [10, 13].

In the current research, culture and sensitivity, cytology and histopathology revealed 12 cases of spinal infection (Table 3) (Figure 2, 3). Among them, eight cases in the thoracic spine and four cases in the lumbar spine. MRI revealed the destruction of the vertebral bodies along with the presence of pre and para-vertebral collections in eight cases. All 12 cases showed a compressed spinal cord due to an epidural component. Four cases were found to be related to cord edema. Mycobacterium tuberculosis was the most common organism responsible for spinal infection causing compressive myelopathy (Table 4). The research conducted by de Roos et al. revealed that mycobacterium tuberculosis was the common organism responsible for spinal infection and thoracolumbar junction was the most often impacted site, which aligns with the current research findings [14].

In the current research, there were eight (16.7%) cases of primary intradural extramedullary tumours. Among these cases, five were identified as neurofibromas and three as meningiomas on histopathology (Table 5, 6). Among the neurofibromas (Figure 4, 5) MRI diagnosed three cases as neurofibromas and two cases equivocal between neurofibroma and meningioma. Among the meningiomas (Figure 6, 7) MRI diagnosed one case as meningioma and two cases equivocal between meningioma and neurofibroma. Neurofibroma was the most common primary intradural extramedullary tumour causing compressive myelopathy. The results of the current research align with the conclusions reported in the research conducted by Abul-Kasim K et al. [5].

The article "Determination of the Efficiency of Magnetic Resonance Imaging in the Evaluation of Compressive Myelopathy" was retracted in 2024. Reasons: plagiarized images; overlap with other authors' work.

In the current research, there were eight (16.7%) cases of spinal metastases on histopathology (Table 6) (Figures 8, 9). Cord compression in all eight patients was caused by intraspinal extradural masses originating from an aberrant portion of the vertebra. It was supported by research performed by Lien et al. [15], wherein 90% of the participants exhibited extradural masses that originated from an aberrant portion of a vertebra. Five (62.5%) of the eight participants had multiple lesions and the dorsal spine was the most frequently affected region in the current research, accounting for 80% of cases. It is similar to the research performed by Lien et al. [15], where 78% of participants had multiple lesions. The predominant primary neoplasms that frequently metastasize to the spine are lung carcinoma, breast carcinoma, and lymphoma [16]. In the current research, there were three cases of carcinoma of the bronchus (Figure 8), three cases of carcinoma of the breast, one case of lymphoma, and one case of carcinoma of the prostate (Figure 9). The results of the current research are similar to the research performed by Lien et al. and Hill et al. [15, 16].

MRI is very useful in deciding the need for surgery and also the type of approach to be followed. MRI also helps in guiding fine needle aspiration cytology (FNAC) whenever there is a dilemma in the diagnosis between the pyogenic and tubercular origin of infection. MRI exhibits high sensitivity and specificity (Table 6) in the identification of extradural and intradural lesions, but occasionally, it might be challenging to distinguish between meningioma and neurofibroma.

There are some limitations inherent in the current research. A limited sample size of patients from a single institution was studied. It was a short-duration study. The current research did not include patients with non-compressive myelopathy and disc herniation. However, the implementation of more comprehensive research endeavours with a larger cohort would yield a more precise depiction of the matter under investigation.

## Conclusions

MRI stands as the gold standard for evaluating soft tissues in the spine and identifying abnormalities in the spinal cord. It excels in evaluating cord edema/contusion, intervertebral disc, and ligament integrity, and serves as the preferred modality for diagnosing spinal trauma, infections, and spinal tumors. While MRI is highly sensitive, the ultimate diagnosis for extramedullary intradural tumors and metastasis still relies on biopsy and histopathological examination. Notably, it remains the sole modality capable of directly visualizing the spinal cord. The current research, utilizing MRI, successfully assessed the spinal cord edema/contusion, intervertebral disc, ligament, and spinal cord integrity in spinal trauma, and spinal infections, characterized the spinal tumors, and classified the tumors based on their locations within the extradural and intradural compartments and established a correlation between MRI findings, intraoperative observations, cytological and histopathological results in operated cases. Therefore, the study concludes that MRI is an extremely reliable, precise, specific, non-intrusive, and radiation-free method for assessing compressive myelopathy.
